The article "Identification of Differentially Expressed Genes Related to Dehydration Resistance in a Highly Drought-Tolerant Pear, Pyrus betulaefolia, as through RNA-Seq" was retracted in 2024. Reasons: concerns about the data; concerns about the results or conclusions.

# Identification of Differentially Expressed Genes Related to Dehydration Resistance in a Highly Drought-Tolerant Pear, *Pyrus betulaefolia*, as through RNA-Seq

**DOI:** 10.1371/journal.pone.0149352

**Published:** 2016-02-22

**Authors:** Kong-Qing Li, Xiao-Yong Xu, Xiao-San Huang

**Affiliations:** 1 College of Rural Development, Nanjing Agricultural University, Nanjing, 210095, China; 2 College of Horticulture, State Key Laboratory of Crop Genetics and Germplasm Enhancement, Nanjing Agricultural University, Nanjing, 210095, China; 3 School of Horticulture and Plant Protection, Yangzhou University, Yangzhou, 225009, China; Key Laboratory of Horticultural Plant Biology (MOE), CHINA

## Abstract

Drought is a major abiotic stress that affects plant growth, development and productivity. Pear is one of the most important deciduous fruit trees in the world, but the mechanisms of drought tolerance in this plant are still unclear. To better understand the molecular basis regarding drought stress response, RNA-seq was performed on samples collected before and after dehydration in *Pyrus betulaefolia*. In total, 19,532 differentially expressed genes (DEGs) were identified. These genes were annotated into 144 Gene Ontology (GO) terms and 18 clusters of orthologous groups (COG) involved in 129 Kyoto Encyclopedia of Genes and Genomes (KEGG) defined pathways. These DEGs comprised 49 (26 up-regulated, 23 down-regulated), 248 (166 up-regulated, 82 down-regulated), 3483 (1295 up-regulated, 2188 down-regulated), 1455 (1065 up-regulated, 390 down-regulated) genes from the 1 h, 3 h and 6 h dehydration-treated samples and a 24 h recovery samples, respectively. RNA-seq was validated by analyzing the expresson patterns of randomly selected 16 DEGs by quantitative real-time PCR. Photosynthesis, signal transduction, innate immune response, protein phosphorylation, response to water, response to biotic stimulus, and plant hormone signal transduction were the most significantly enriched GO categories amongst the DEGs. A total of 637 transcription factors were shown to be dehydration responsive. In addition, a number of genes involved in the metabolism and signaling of hormones were significantly affected by the dehydration stress. This dataset provides valuable information regarding the *Pyrus betulaefolia* transcriptome changes in response to dehydration and may promote identification and functional analysis of potential genes that could be used for improving drought tolerance via genetic engineering of non-model, but economically-important, perennial species.

## Introduction

As sessile organisms, plants are frequently threatened by drought, which detrimentally affects growth, development, productivity and geographic distribution [1]. Plants have developed many sophisticated mechanisms to adapt or survive under drought stress. Elucidating the molecular mechanisms that regulate drought tolerance is critical if plant growth and productivity under drought conditions is to be improved. Emerging evidences have shown that plants do not passively accept adverse conditions, but cope with it actively through generic drought signal perception and transduction, which leads to a range of stress related genes alterations that protect them from stress [2].

Previous reports have indicated that stress signaling cascades encompass a large number of stress-responsive genes, which can be generally classified into two major groups based on the functions of their products, effector molecules or regulator molecules. Products of the first group fucntion directly in protecting cells against damage derived from stresses and sustaining cell viability, such as osmolyte biosynthetic enzymes, antioxidant proteins, chaperones and late embryogenesis abundant (LEA) proteins [2–5]. The second group is composed of regulatory proteins, such as transcription factors (TFs), protein phosphatases and protein kinases [2]. Among these stress-related transcription factors, members of the AP2/EREPB, bZIP, WRKY and MYB proteins have been well characterized for their roles in the regulation of drought tolerance [6–9]. These genes constitute a delicate network that plays a key role in combating abiotic stress. A large number of genes are expressed under abiotic stress conditions, which suggests that the abiotic stress responses are more complex than was previously thought. Furthermore, there has been some difficulty in developing a clear-cut network for abiotic stress responses. Although many molecular components responsive to drought stress have been identified in many model plants, the highly complex and interconnected nature of the network is still not understood. Furthermore, it is well known that molecular responses may differ between model plants and non-model plants, although a few parts of the response pathways may be the same. Therefore, it is important to identify transcriptional changes in non-model plants during drought stress so that the molecular elements that are specific to non-model plants can be identified.

Previous researchers tended to clone and characterize a single gene involved in the stress response. However, this is a piecemeal strategy and contributes little to a comprehensive understanding of the defense-related transcriptome that is controlled by quantitative mechanisms [10]. To extend the list of candidates of interest, high-throughput techniques have been widely applied to further understanding of the molecular mechanisms underlying drought stress. Genome-wide expression profiling of plants under drought stress has been reported for many plant species, including tomato [11], rice [12], barley [13], cotton [14], maize [15], sorghum [16] and *Arabidopsis* [17, 18]. Although significant progress has been made over the past decade into identifying the networks affected by drought stress, there is still little information available about the network dynamics involved in pear drought resistance.

Pear is the one of the most widespread fruit in the world and has considerable economic and health value. Many wild relatives of cultivated pear exist and they have different degrees of tolerance to abiotic stress. *Pyrus betulaefolia*, an important rootstock for pear, is drought tolerant, which makes it a good source of valuable drought tolerance genes [19, 20]. Furthermore, genomic information for pear is currently available, and RNA-Seq has become more efficient, less costly and more sensitive [21, 22]. In this study, RNA-Seq data were generated to compare the gene expression patterns during different dehydration states. The gene expression profiles will provide valuable insights into the mechanisms underlying drought resistance in pear.

## Materials and Methods

### Plant materials and dehydration treatment

Pear plants were grown in the seedling beds at National Center of Pear Engineering Technology Research, Nanjing Agricultural University. Three-month-old plants were used in this study. Uniform and healthy plants were inserted into a beaker containing distilled water, which were kept in a growth chamber at 26°C with a 16 h light/8 h dark photoperiod for 2 d before exposure to the dehydration treatment. Then seedlings were put on clean filter papers (90 x 90 mm) and allowed to dry for 0, 1, 3 and 6 h in an ambient environment at 26°C, followed by recovery in water at 26°C for 24 h. The leaves were independently harvested at the designated dehydration time points and then immediately placed in liquid nitrogen, and stored at –80°C until they were used for RNA extraction.

### Illumina sequencing and data analysis

The total RNA isolation and Solexa/Illumina sequencing was done according to the published paper [23]. The raw sequence data analysis and base calling were produced by the Illumina instrument software Analyzer at BGI-Shenzhen. The remaining high quality clean sequencing reads were mapped onto the pear genome reference [24] to identify continuous gene regions using SOAP aligner/SOAP2 [25]. Only two mismatches were allowed. Unique mapped reads were used for further analysis. For gene expression level analysis, RPKM (reads per kb per million reads) was used [26]. To identify differentially expressed genes (DEGs), read counts for each gene were calculated. Then we model the read counts as Poisson distributed [27]. DEGs were identified requiring FDR ≤ 0.001 and an absolute value of log_2_ (fold-change) ≥ 1.

Genes with similar expression patterns are usually functionally correlated. We performed a cluster analysis on the gene expression patterns using cluster software [28] and Java Treeview [29] software. In the gene expression profiling analysis, InterPro domains [30] were annotated by InterProScan Release 36.0 [31] and functional assignments were mapped onto GO terms [32]. GO enrichment analysis were constructed using WEGO [33]. Significantly enriched Kyoto Encyclopedia of Genes and Genomes (KEGG) pathways were identified according to the P values and enrichment factors [34]. Using a BLAST search against the KEGG database and then mapped onto KEGG pathways.

### Cluster analysis

For each gene, RPKM expression values were normalized to values between -1.0 and 1.0 by multiplying by a scale factor, which made the sum of the squares for the time point values equal to 1.0. The normalized expression values for each transcript were then centered on zero by subtracting the mean of the values from each data point. Clustering was carried out by hclust function in R (http://www.r-project.org/) using a distance matrix representing the RPKM level profiles of the genes across the five time points. The tree produced by the clustering process was cut into several groups by the cutree function in R. Maximum number of clusters was set to 20.

### Gene expression analysis by quantitative real-time PCR

To validate the expression patterns reveals by digital transcript abundance measurements results, sixteen DEGs were randomly selected and analyzed using quantitative real-time PCR. Primers for 16 DEGs were designed using Primer 5 software based on the target genes and listed in S11 File. Total RNA was treated with Dnase I to remove genomic DNA contamination, and then about 1μg of total RNA was used cDNA synthesis by the ReverTra Ace-αFirst Strand cDNA Synthesis Kit (TOYOBO, TOYOBO Biotech Co. Ltd, Japan) following the manufacturer’s instructions. The 10 μL qPCR solutions contained 5 μL of SYBR^®^ Green Premix kit (TaKaRa Biotechnology. Dalian, China), 0.25 μM forward and 0.25 μM reverse primers, and 50 ng cDNA templates. All reactions were run as duplicates in 96-well plates. The quadruple qPCR reactions were performed on a Lightcycle-480 (Roche) using the following cycle regime: 50°C/2 min, 95°C/10 min, followed by 40 cycles of 95°C/15 s, and 58°C/1 min. The *Tubulin* gene (AB239681) was amplified in parallel as an internal reference gene. The relative expression levels of the amplified products were calculated using the 2^-ΔΔCt^ method [35]. Four technical replicates were used for each sample and the data are shown as means ± standard errors (SE) (n = 3). The source of variation resulted from the technical errors, such as operational approach, equipment and reagent. The primer sequences used for qPCR are listed are listed in S11 File.

## Results and Discussion

### Electrolyte leakage and relative water content during dehydration

In order to investigate the effect of dehydration on pear, young seedlings were dehydrated for 0, 1, 3, 6 h in an ambient environment at 26°C, followed by recovery in the water at 26°C for 24 h (Fig 1). Seedling electrolyte leakage (EL) was measured. Significantly higher EL was observed during dehydration for 6 h than at any other time point. The survival rate of the plants dehydrated for 6 h was 42% (Fig 1F). The decrease of relative water content (RWC) in the leaves was slow over the first hour of dehydration in an ambient environment but accelerated at the 3 and 6 h time points. The RWC of the dehydrated plants after 6 h was lower than it was at the other time points, except for after recovery in the water for 24 h (Fig 1F). The net photosynthetic rate (*P*_n_), stomatal conductance (*G*_s_) and transpiration rate (*T*_r_) of *Pyrus betulaefolia* were lower at 6 h than for any of the other time points at 1000 mol·m^-2^·s^-1^ light intensity. In this study, we also monitored the water potential during the process of dehydration, the result was shown as (S1 Fig). These results agree with earlier reports that drought significantly damages self-repair mechanisms and physiological metabolism [36–39].

**Fig 1:** Time-course fresh water loss of *Pyrus betulaefolia* seedling during dehydration for 0, 1, 3 and 6 h in an ambient environment at 26°C, followed by recovery in water at 26°C for 24 h. (A-E). Electrolyte leakage and relative water content (RWC) analysis of *Pyrus betulaefolia* leaves. (F). Content of photosynthetic rate (*Pn*) (G); content of stomatal conductance (*Gs*) (H); content of transpiration rate (*Tr*) (I).

### Statistics of read mapping

In this study, we performed an RNA-Seq analysis of the *Pyrus betulaefolia* digital transcript abundance measurements using Illumina-based 2 × 90 bp paired-end reads sequencing. Illumina, a widely used NGS platform for transcriptome assembly, produces relatively shorter reads but generates higher transcriptome coverage at lower expenses compared with other platforms [40]. In total, five RNA-Seq libraries were sequenced from *Pyrus betulaefolia* shoots dehydrated for 0, 1, 3 or 6 h in an ambient environment and then left to recover for 24 h in water. The number of reads for each library ranged from 11.7 to 12.6 million. A total of 11,959,230 raw reads were obtained from D0, 11,784,133 from D1, 12,643,252 from D3, 12,388,234 from D6, 11,957,932 from DH24. We filtering out the low quality reads, reads where the percentage of unknown bases (N) was greater than 10%, and adaptor sequences. Finally, this generated 11,403,704; 11,260,699; 12,317,953; 11,922,934; 11,408,119 clean reads with 49 bp reads for the 0, 1, 3, 6, dehydration time points and the 24 h recovery time point. The average number of clean reads produced per library was 11.6 million. The total number of mapped reads per library ranged from 7.9 to 8.6 million and the percentage of these mapped reads ranged from 70% to 71% (Table 1).

**Table 1:** Summary of read numbers based on the RNA-Seq data from *Pyrus betulaefolia* pear during dehydration.

Summary	D 0	D 1	D 3	D 6	DH 24
Total clean Reads	11,403,704	11,260,699	12,317,953	11,922,934	11,408,119
Total Mapped Reads	8,027,870	7,923,533	8,647,506	8,577,648	8,049,552
Total Mapped Reads/Total clean Reads	70.40%	70.36%	70.20%	71.94%	70.56%
Perfect Match Reads	4,608,911	4,588,977	5,021,477	4,940,970	4,651,945
Perfect Match Reads/Total clean Reads	40.42%	40.75%	40.77%	41.44%	40.78%
≤2 bp Mismatch Reads	3,418,959	3,334,556	3,626,029	3,636,678	3,397,607
≤2 bp Mismatch Reads/Total clean Reads	29.98%	29.61%	29.44%	30.50%	29.78%
Unique Match Reads	6,132,881	6,068,845	6,132,881	6,132,881	6,132,881
Unique Match Reads/Total clean Reads	53.78%	53.89%	52.48%	55.71%	52.97%
Multi-Position Match Reads	1,894,989	1,854,688	2,182,942	1,935,434	2,006,133
Multi-Position Match Reads/Total clean Reads	16.62%	16.62%	16.62%	16.62%	16.62%
Total-Unmapped Reads	3,375,834	3,337,166	3,670,447	3,345,286	3,358,567
Total-Unmapped Reads/Total clean Reads	29.60%	29.64%	29.80%	28.06%	29.44%

In this study, reads of RNA-Seq data were mapped to the assembled pear genome for ‘Dangshansuli’ [24]. A saturation analysis was performed to determine if the number of the detected genes increased in proportion to the sequencing effort. The saturation trend showed that the number of detected genes almost stopped increasing when the number of reads reached 2 million (data not shown). If the randomness is poor for specific gene region, then this will directly affect subsequent bioinformatics analysis. Therefore the randomness of the RNA-seq data was evaluated by analyzing the distribution of reads matching the reference genes [41]. The results showed that the randomness of the reads was so good that the reads in every position would be evenly distributed (data not shown). Heterogeneity and redundancy are two significant characteristics of mRNA expression levels. Therefore, the normality of the RNA-Seq analysis was evaluated by analyzing the distribution of the unique mapped reads. S2 Fig shows that the distribution of the unique mapped reads over different read abundance categories showed the same patterns for all five RNA-Seq libraries. Taken together, these results were also suggested that our RNA-seq data of *Pyrus betulaefolia* represents a valuable digital transcript abundance measurements resource for gene discovery and functional analysis, which was in agreement with previous report [11, 13, 21, 23].

### Differentially expressed genes in the libraries

It has been well documented that plants can enhance their drought tolerance by modulating gene transcription, and examples of gene induction and repression in response to drought have been reported [11, 42]. In this study, differences in gene expression during dehydration treatment were analyzed, and the DEGs were identified by pairwise comparisons of the five libraries, i.e. D0 vs. D1, D0 vs. D3, D0 vs. D6, D0 vs. DH24, D1 vs. D3, D vs. D6, D1 vs. DH24, D3 vs. D6, D3 vs. DH24 and D6 vs. DH24 (Fig 2A), which resulted in ten pairs of comparisons. Among these comparisons, we found that between 374 and 6866 genes were significantly differentially expressed, depending on the library, and the average number was 3,777. The differential expression patterns for the libraries revealed that the largest number of differentially expressed genes occurred between D0 and D6. A total of 6866 genes were significantly differentially expressed between these two libraries. Of these genes, 3060 genes were up-regulated and 3806 genes were down-regulated. The second largest number of differentially-expressed genes occurred between D1 vs. D6. A total number of 6,150 DEGs were detected between the D1 and D6 libraries, with 3087 being up-regulated and 3063 down-regulated. The third largest number of DEGs occurred in the D6 vs. DH24 comparison, followed by D3 vs. D6, D1 vs. D3, D1 vs. DH24, D3 vs. DH24, D0 vs. D3, D1 vs. D3, D0 vs. D1. The results are consistent with the results reported by Huang et al. (2013), Ning et al. (2010), Gong et al. (2010), whose data showed that on exposure to different stresses, many stress related genes were induced by stress treatments that lasted for varying lengths of time [21, 43, 44]. One of the explanations for this might be that plants do not passively accept environmental stresses, but respond actively through the perception of a stress signal, which then induces the expression of a large number of stress related genes that protect the plant against stress damage [13, 36]. To further survey the genes that were transcriptionally highly expressed during specific stages of dehydration, we investigated the genes that were up-regulated at a single time point compared with their expression levels at any other time point. There were 1516 relatively highly expressed genes that showed a more than twofold change in expression at a single stage compared to all other stages (S1 File). These genes are called stage specific up-regulated genes (SSRG) in this paper. After the plants had been dehydrated for 1 h, ten genes showed a more than twofold change in expression, compared to the other time points. Two of these SSRG genes coded for 70 kD heat shock proteins (Hsp70s), which are an important part of a cell’s protein folding mechanism, and help to protect cells from stress [45]. Five genes were related to protein folding, which indicated that the protein folding mechanism was the main process that responded to drought stress at this point. After 3 h, 53 SSRGs were observed to be enriched in the GO terms “apoptosis” and "protein phosphorylation" (Table 2). After 6 h, the number of SSRGs significantly increased. A total of 992 SSRGs were detected with the enriched GO terms of “regulation of transcription”, “NA-dependent”, “response to biotic stimulus”, “cell wall macromolecule catabolic process” etc. After the rehydration recovery period in water, there were 457 genes that were more highly expressed than at any other stage. The up-regulated transcription of the genes mentioned above suggested that they played an important role in biological processes at specific stages during dehydration. During the early stage of dehydration stress, protein folding is important, and then apoptosis and protein phosphorylation began to respond to stress after 3 h of treatment. Many genes were highly expressed after 6 h, including some transcription factors and stress related genes (S2 File). When the plants had recovered in water, other highly expressed genes seemed to play a specific role in recovery, which was in agreement with previous report [13, 37, 43].

**Fig 2:** Differentially expressed genes between different libraries. Up-regulated (red) and down-regulated (green) genes were quantified (A). The ten comparison results are shown. Venn diagram showing the differentially expressed genes at each of the five time points associated with drought stress. (B) Up-regulated genes. (C) Down-regulated genes.

**Table 2:** Over-represented GO terms for specific highly expressed genes at a given time point compared to the other time points.

Stage	GO description	Number of genes	P value
D1.UP	protein folding	5/250	7.1E-08
	response to stress	2/659	4.8E-02
D3.UP	apoptosis	7/296	1.6E-04
	protein phosphorylation	9/1429	4.4E-02
	innate immune response	3/104	1.8E-02
D6.UP	regulation of transcription, DNA-dependent	48/679	2.2E-02
	response to biotic stimulus	8/48	2.6E-02
	response to water	4/11	2.5E-02
	pentose-phosphate shunt	4/12	2.6E-02
	aromatic amino acid family metabolic process	7/38	2.6E-02
	cell wall macromolecule catabolic process	7/31	1.6E-02
D6.DOWN	photosynthesis, light harvesting	14/28	1.8E-09
	pigment biosynthetic process	6/22	4.6E-02
	L-arabinose metabolic process	3/3	1.2E-02

We analyzed genes that were only differentially expressed at a single time point to investigate genes that are transcriptionally regulated at specific time points under water deficit conditions. We found that 26, 166, 1295 and 1065 of the DEGs were significantly up-regulated only at D1, D3, D6 and DH24, respectively (Fig 2B). In contrast, 23, 82, 2188 and 390 genes were only significantly down-regulated at D1, D3, D6 and DH24, respectively (Fig 2C). We also have added the analysis on each stage (D1, D3 and D6) specific down-regulated genes compared with DH24, the data are shown in S3, S4, S5 and S6 Files. In addition, we have added the analysis on 5 stages common differentially expression genes. There were 70 genes common up-regulated, and 78 genes are common down-regulated (S7 and S8 Files). These data indicate that DEGs display noticeable differences in their dehydration response at the transcriptional level, and that these differences depend on the dehydration state of the plant, which was in agreement with previous report [11, 13].

### Functional annotation of differentially expressed genes

BLAST analysis and GO term annotation were performed to improve our understanding of the functions of these specifically regulated genes. We used GO term enrichment analysis to gain more insights into these genes. It is an efficient strategy for analyzing the representation of genes in different categories because it compares gene expression profiles to the background profile [46]. GO term enrichment analysis annotated approximately 19,532 sequences and categorized them into three main categories: biological process, cellular component and molecular function. The sequences were subsequently categorized into 40 GO functional groups (Fig 3). In the biological process category, the DEGs were further classified into four major groups: metabolic processes, cellular processes, response to stimulus and biological regulation. In the molecular function category, the genes were further classified into seven major groups: catalytic activity, binding, transporter activity, molecular transducer activity, transporter activity, enzyme regulation and nucleic acid binding transcription factor activity. The cellular component category was further classified into cell, cell part, membrane, organelle and membrane part. These results demonstrated that DEGs that had binding, transport, molecular transduction, transcription regulation and enzyme regulation functions were important during drought stress, which was in agreement with previous report [11, 21].

**Fig 3:** GO categories for the genes identified. Y-axis (left) represents the percentage of genes identified in this study; Y-axis (right) represents the actual gene number. The genes were annotated into three main categories: biological process, cellular component and molecular function (X-axis).

Significantly enriched Kyoto Encyclopedia of Genes and Genomes (KEGG) pathways were identified according to the P values and enrichment factors. Using a BLAST search against the KEGG database showed that there were 19,532 genes that mapped onto KEGG pathways. As shown in S9 File, a total of 129 KEGG pathways were observed to be significantly overrepresented during dehydration. The genes that correlated with drought were mainly involved in photosynthesis, plant hormone signal transduction, cell wall modification, transcriptional regulation and drought metabolism, and were selected for subsequent analysis. The present results were consistent with the overall biochemical pathways that are known to be active during drought stress [11]. In addition, several other biological processes that have not previously been reported to be associated with drought, such as cell process, biological regulation, and metabolic process, also dramatically changed during drought stress. These might be novel genes that are relevant to the drought process in *Pyrus betulaefolia*, which was in agreement with previous report [43, 47].

### An overview of the gene expression profiles, gene ontology enrichment results and KEGG pathways present during dehydration treatment

To investigate the co-expressed genes during drought stress, we applied statistical clustering to all the genes that were differentially expressed in at least one drought stage compared to the control (Fig 4). This clustering approach classifies genes using the pool of differentially regulated genes that exhibited similar patterns of expression over the five stages, regardless of the absolute level of expression. We detected 18 clusters of regulated genes, comprising of 8538 genes that showed some degree of differential expression (Fig 4). The largest group (Cluster 1) included 2335 genes (27.3%) that began to decrease progressively 3 h after dehydration treatment, but maintained a stable expression level during the last two stages. The second largest group (Cluster 3) contained 2008 genes (23.5%) that began to accumulate 1 h after dehydration, and increased progressively until they reached their highest level at 6 h. The third largest group (Cluster 5) contained 1044 genes (12.2%) whose expression decreased continuously up to the 6 h time point, and then increased progressively until they reached their highest level at DH24. The fourth largest group (Cluster 6) contained 1030 genes (12.1%) whose expression did not change notably at the beginning, except for a slight decrease at 6 h of dehydration treatment, and then increased progressively until the end at DH24. The fifth largest group (Cluster 8) contained 838 genes (9.8%) whose transcript level increased progressively under dehydration stress until they reached their highest level at 6 h, and then slightly decreased until the end at DH24. The sixth largest group (Cluster 11) contained 116 genes (1.4%) whose expression increased continuously under dehydration stress until they reached their highest level at 6 h, and then decreased progressively until DH24, which was in agreement with previous report [36, 37].

**Fig 4:** Clustering and gene ontology enrichment of regulated genes. Genes displaying some degree of regulation were clustered using Hierarchical Clustering. A description of the expression pattern and the number of transcripts belonging to the cluster form the title of each chart. Expression values were normalized and scaled to between –1.0 and 1.0 (Y-axis). Enriched “Biological Process” GO terms, generated in BinGO are listed at the bottom of each cluster. For Clusters 12, 13, 14, 16 and 18, no over-represented “Biological Process” terms were detected. The number of genes associated with an over-represented GO term in the cluster and the number of genes associated with the same GO term in the Pyrus transcriptome are shown in parentheses. Specific genes belonging to each cluster can be found in S3 File. 2 (D1), 3 (D3), 4, (D6), 5 (DH24).

In order to produce a global description of the biological processes enriched in each cluster of similarly regulated genes, we generated an overview of gene ontology (GO) terms using BinGO. The GO term “photosynthesis” was enriched in Cluster 1, which indicated that photosynthesis decreased when the plant responded to water deficit stress. The “innate immune response” biological process was detected in Clusters 2 and 11, whose genes were highly expressed at D3 or D6, but had returned to control levels at DH24. The “response to stimulus” and “response to water” biological processes were also represented in Cluster 3, The transcript levels of the genes in these groups increased progressively under dehydration stress and reached their highest level at 6 h, and then decreased progressively after the plants had been allowed to recover for 24 h. Cluster 5 enriched GO terms, such as “regulation of cellular protein” and “metabolic process”, contained up-regulated genes. These results suggested that genes with significantly up-regulated expressions under these GO terms played key roles in the response to dehydration stress, which was in agreement with previous report [43, 47, 48].

We generated an overview of the metabolic pathways using KEGG pathway analysis (http://www.genome.jp/kegg/) so that a global description of enriched metabolic pathways in each cluster of similar genes could be produced. We also found other important metabolic pathways that had been enriched in some clusters and were related to drought stress (S2 File). “Plant hormone signal transduction” and “photosynthesis” was found to be enriched in Cluster 1, which showed that photosynthesis pathway activity decreased when plants were exposed to dehydration stress. These results agreed with earlier reports that photosynthesis is a primary biosynthetic pathway that restricts the normal function of other metabolic pathways, such as nitrogen fixation [11, 49, 50]. The metabolic “MAPK signaling pathway” was classified into Cluster 3 and Cluster 15. Previous studies have extensively emphasized the role of the MAPK signaling pathway in abiotic stress tolerance [38, 44, 51, 52].

### Metabolic changes of hormone in response to the dehydration

In order to investigate the metabolic changes after dehydration stress, we used MapMan to dissect the detailed metabolism in pear. At D1 and D3, we can observed that some of mebabolism have been changes, including genes including genes involved in cell wall, lipids, etc. We also observed the most metabolic changes at D6 (S3, S4, S5 and S6 Figs). Plant utilize hormones to regulate and coordinate growth and stress tolerance to survive or escape from stress. These hormones can act in the upstream of dehydration response and trigger hormone signal pathway. So here we mainly focus on metabolic changes of Abscisic acid (ABA) and gibberellin (GA).

Abscisic acid (ABA) is an important phytohormone in the dehydration-stress response in plant. Its metabolic changes are one of the determinants of endogenous ABA levels and control diverse stress response. In our results, we observed *PbNCED3* were induced at 1 h and kept a higher expression level at 3 h and 6 h. After recovery in the water for 24 h, the expression was down-regulated. This gene encodes an epoxy carotenoid dioxygenase, a key enzyme in the biosynthesis of abscisic acid. *AtNCED3* gene is strongly induced by drought stress, and the *nced3* mutant lacks drought-responsive ABA accumulation [53]. The induction of *AtNCED3* occurs in the early stages of the response to dehydration stress [54]. In our study, *PbNCED3* was also induced at very early stage (Fig 5A).

**Fig 5:** Expression patterns of genes involved in ABA and GA metabolism.

In pear, *PbCYP707A3* showed similar expression pattern with *PbNCED3* (Fig 5B). The *cyp707a3* mutant plants exhibited both exaggerated ABA-inducible gene expression and enhanced drought tolerance [55]. *CYP707A3* encodes a major ABA 8'-hydroxylase and involves in dehydration and rehydration response in *Arabidopsis* [55]. These results indicate that the response of the ABA metabolism pathway towards drought stress is a conserved mechanisms between *Arabidopsis* and pear.

We found that *PbCYP88A3* were induced under drought stress in pear (Fig 5C). *PbCYP88A3* encodes an ent-kaurenoic acid hydroxylase. Ent-kaurenoic acid hydroxylase is an important enzyme in GA biosynthesis. After drought stress, ent-kaurenoic acid hydroxylase was found to be down-regulated. GA 2-oxidase (GA2ox) genes encode GA-inactivating enzymes [56]. GA deactivation is an important point of control in the reduction of bioactive GA levels in response to stress. Decreased level of bioactive GA levels may be a results of growth inhibition after dehydration in pear (Fig 5D).

### Phytohormone signal transduction under dehydration stress

In our work, the digital transcript abundance measurements data showed that the transcript levels of genes involved in signal transduction pathways related to plant hormone were chaged within 1 h of dehydration treatment. Furthermore, a large numbers of genes related to hormone pathways showed modifys in transcript levels over the 6 h of the dehydration, demostratting a important role of the these pathways in conferring *Pyrus betulaefolia* response to the dehydration. ABA is a major phytohormone that regulates a broad range of plant traits and is important for adaptation to environmental conditions [56, 57]. It has been suggested that ABA can bind to the PYR/PYL/RCAR family of START domain-containing soluble receptors [58, 59]. The binding causes the receptors to bind and inhibit the activities of the type A protein phosphatase 2Cs (PP2Cs). Intersetingly, in this study, we noticed that a PYL gene was up-regulated by approximately 7–50 folds after 3 and 6 h of dehydration treatment. Up-regulation of the PYL gene implies that synthesis of ABA might be elevated in *Pyrus betulaefolia* under dehydration. In addition, we also detected the up-regulated expression of PP2C by approximately 5.6–9.7 folds after 3 and 6 h of dehydration treatment, a key component in the ABA signaling pathway. This result is consistent with studies of *P*. *euphratica* and *A*. *thaliana* [11, 60]. So, whether and how ABA mediated signaling pathway is involved in the dehydration responses of *Pyrus betulaefolia* remains to be further illustrated.

### Classification of the transcription factors into clusters

Numerous families of TFs are known to orchestrate the signals that are transduced when plants are challenged with various abiotic stresses, including the MYB, AP2/ EREBP, WRKY, NAC, MYC and bHLH families, and individual members have been revealed to promote or suppress abiotic stress responses [6, 8, 43, 61–64]. In the current study, our digital transcript abundance measurement results showed that 2353 TFs were annotated as putative transcription factors in the pear genome. Among these, 637 (27.1%) were found to be induced either at a given time point or during the whole course of the dehydration treatment. These TFs were distributed across the above 18 clusters and classified into five major groups according to their putative DNA binding domains (S10 File).

The first largest group of the dehydration-inducible TFs belonged to the MYB family, which contained 72 MYB genes that were differentially expressed and classified into different clusters based on their expression patterns, among which 23, 6, 17, 1, 6, 4, 5, 6, 2 and 2 MYB transcription factors were identified in Cluster 1, Cluster 2, Cluster 3, Cluster 4, Cluster 5, Cluster 6, Cluster 7, Cluster 8, Cluster 11 and Cluster 16, respectively (S10 File). Interestingly, Clusters 2, 3, 8, 11 and 16 were induced by the drought treatment. In other words, approximately 33 MYB transcription factors were up-regulated under dehydration stress. The present data corroborated earlier work which had suggested that MYB family transcription factors were involved in stress responses [6, 65].

The second group of induced transcription factors contained factors from the basic helix-loop-helix (bHLH) family. A total of 57 bHLH genes were identified as drought-responsive genes in this study. Approximately 24, 2, 17, 1, 5, 3, 3, 1 and 1 bHLH transcription factors were identified in Cluster 1, Cluster 2, Cluster 3, Cluster 4, Cluster 5, Cluster 6, Cluster 8, Cluster 12 and Cluster 17, respectively (S10 File). Cluster 3 and Cluster 8 genes, whose transcription levels increased progressively under dehydration stress, contained 20 bHLH transcription factors. In addition, one bHLH transcription factor was up-regulated at D1, 11 bHLH novel genes were up-regulated at D3, 11 bHLH novel genes were up-regulated at D6, and three bHLH novel genes were up-regulated at DH24. Our data corroborates earlier research that had suggested that the bHLH genes were involved in ABA response regulation under stress conditions [64, 66].

The third group contained 45 WRKY genes that were induced by dehydration treatment. In this study, a total of 45 WRKY transcription factors were differentially expressed, and approximately 4, 6, 23, 2, 3, 5, 1 and 1 WRKY transcription factors were identified in Cluster 1, Cluster 2, Cluster 3, Cluster 5, Cluster 6, Cluster 8, Cluster 9 and Cluster 11, respectively (S10 File). Moreover, one WRKY transcription factor was induced at D1, 23 WRKY novel genes were up-regulated at D3, nine WRKY novel genes were up-regulated at D6, and four novel genes were up-regulated at DH24. These results agree with earlier reports that WRKY transcription factors play important roles in regulating drought and other abiotic stress responses [67, 68].

The fourth group contained NAC family genes, and a total of 39 genes belonging to this family were identified in this study. Among them, approximately 3, 2, 20, 3, 4, 6 and 1 NAC transcription factors were classified into Cluster 1, Cluster 2, Cluster 3, Cluster 4, Cluster 5, Cluster 6, Cluster 8, Cluster 9 and Cluster 11, respectively (S10 File). In addition, three NAC transcription factors were induced at D1, 12 novel NAC genes were up-regulated at D3, 13 novel NAC genes were up-regulated genes at D6, and four novel NAC genes were up-regulated at DH24. These results agreed with earlier reports that suggested that NAC genes played significant roles in plant tolerance to various environmental stresses [63, 69].

The fifth group contained HSF family genes. A total of 15 HSF genes were induced by dehydration treatment in this study. Of these, 10, 1 and 4 HSF transcription factors were classified into Cluster 3, Cluster 11 and Cluster 15, respectively (S10 File). Furthermore, four HSF transcription factors were induced at D1, six novel HSF genes were up-regulated at D3, and seven novel HSF genes were up-regulated at D6. However, there was only one novel HSF up-regulated at DH24. Several earlier studies have demonstrated that HSF family genes are regulators that prevent the accumulation of damaged proteins and maintain cellular homeostasis [70, 71], but whether they work, independently or synergistically, to promote drought tolerance of *Pyrus betulaefolia* remains to be determined.

### Validation of DEG-based gene expression

To validate the reliability of the drought responsive gene expression profiles for DEG, 16 genes were confirmed by quantitative real-time PCR using gene-specific primers (S11 File). These selected genes encoded dehydrin 5, dehydrin 2, dehydrin 4, dehydrin 1, heat stress transcription factor A-3-like, ethylene response factor 3, WRKY transcription factor, late embryogenesis abundant protein D-29, putative transcription factor bHLH041, CML13, PP2C, DREB6 and WRKY29. As shown in Fig 6, it is evident that the expression patterns of the selected drought responsive genes produced by quantitative real—time PCR were largely consistent with the DEG data, despite the difference in the absolute fold change between the two methods. These results agreed with earlier reports that suggested that these selected genes played significant roles in plant tolerance to various environmental stresses [5, 8, 22, 57, 59, 68, 70, 72, 73]. It also showed that there is a high degree of correlation in expressional patterns between qPCR and RNA-Seq. In addition, The PCR efficiency (E) of each gene were ranked from 95.7% to 105.5%, the correlation coefficients (R^2^) was between 0.996 to 1.000. The result indicated that the primer for quantitative real-time PCR of each gene was appropriate (S11 File). This suggested that the results from this preliminary DEG data analysis were reliable, which was in agreement with previous report [21, 74]. In addition, it also provides a basis for further investigation into the functions of these drought genes in the future.

**Fig 6:** Quantitative RT-PCR validation of differential gene expression during dehydration. The left Y-axis indicates the gene expression levels calculated by the RPKM method. The right Y-axis indicates the relative gene expression levels.

## Conclusions

The transcriptome data for *Pyrus betulaefolia*, obtained by RNA-Seq, was used to identify and annotate a large number of DEGs involved in dehydration stress, which provides an excellent platform for future genetic and functional genomic research. Genes related to drought tolerance and their expression profiles at four different dehydration stages and at one recovery stage were analyzed further. This offered new insights into the molecular mechanisms underlying pear drought tolerance. The up-regulated DEGs included some previously reported genes (e.g. NAC, DREB, bHLH and MYB) and some new genes (e.g. cytochrome P450, ERF1B and PYL) that are thought to be related to drought tolerance. In addition, a number of candidate target genes that could be used in future functional studies of the drought stress process were obtained. Taken together, in this study, we found metabolic changes of ABA and GA in pear. These changes worked as upstream of drought response and then leaded hormone signal changes. Hormone signal changes further caused TF expression changes and drought response in pear (S7 Fig). The data presented here gives an insight into the molecular changes underlying the drought process in *Pyrus betulaefolia*, and the results can be used as a reference for identifying candidate genes that hold great potential for genetic engineering and for the creation of novel germplasms with enhanced drought stress tolerance.

## Supporting Information

S1 Fig Water potential during the process of dehydration. (JPG)

S2 Fig Percent coverage represents the percentage of unigenes mapped in our transcriptome data that showed a five-fold increase in expression during dehydration. Gene coverage is the percentage of a gene covered by reads. This value is the ratio of the number of bases in a gene covered by unique mapping reads to the total number of bases in that gene. The distribution of unique reads over different read abundance categories show similar patterns for all five RNA-Seq libraries.
(TIF)

S3 Fig DEGs between D0 and D1 in major metabolic pathway using MapMan. (JPG)

S4 Fig DEGs between D0 and D3 in major metabolic pathway using MapMan. (JPG)

S5 Fig DEGs between D0 and D6 in major metabolic pathway using MapMan. (JPG)

S6 Fig DEGs between D0 and DH24 in major metabolic pathway using MapMan. (JPG)

S7 Fig Model for drought response in pear. (TIF)

S1 File Best hit counterparts in other plant species of the genes specifically up-regulated in a stage compared with other stages (DOCX)

S2 File Significantly enriched pathway in KEGG in clusters. (XLSX)

S3 File D0 stage specific down-regulated genes compared with DH24. (XLSX)

S4 File D1 stage specific down-regulated genes compared with DH24. (XLSX)

S5 File D3 stage specific down-regulated genes compared with DH24. (XLSX)

S6 File D6 stage specific down-regulated genes compared with DH24. (XLSX)

S7 File Common up-regulated genes in D1, D3, D6 and DH24. (XLSX)

S8 File Common down-regulated genes in D1, D3, D6 and DH24. (XLSX)

S9 File Significantly enriched Kyoto Encyclopedia of Genes and Genomes (KEGG) terms. (XLS)

S10 File List of TFs in each cluster. (XLSX)

S11 File Primers for sixteen DEGs were designed using Primer5 software based on the target genes. (DOCX)

## References

[1] AswathCR, KimSH, MoSY, KimDH. Transgenic plants of creeping bent grass harboring the stress inducible gene, 9-cis-epoxycarotenoid dioxygenase, are highly tolerant to drought and NaCl stress. Plant growth regulation. 2005;47(2–3):129–39. 10.1007/s10725-005-3380-6

[2] ShinozakiK, Yamaguchi-ShinozakiK. Gene networks involved in drought stress response and tolerance. Journal of experimental botany. 2007;58(2):221–7. 10.1093/jxb/erl164 .17075077

[3] BaillyC, AudigierC, LadonneF, WagnerMH, CosteF, CorbineauF, et al Changes in oligosaccharide content and antioxidant enzyme activities in developing bean seeds as related to acquisition of drying tolerance and seed quality. Journal of experimental botany. 2001;52(357):701–8. .1141320610.1093/jexbot/52.357.701

[4] BretonG, DanylukJ, CharronJBF, SarhanF. Expression profiling and bioinformatic analyses of a novel stress-regulated multispanning transmembrane protein family from cereals and Arabidopsis. Plant physiology. 2003;132(1):64–74. 10.1104/pp.102.015255 .12746512PMC166952

[5] WangYC, JiangJ, ZhaoX, LiuGF, YangCP, ZhanLP. A novel LEA gene from Tamarix androssowii confers drought tolerance in transgenic tobacco. Plant Science. 2006;171(6):655–62. 10.1016/j.plantsci.2006.06.011

[6] AbeH, YamaguchiShinozakiK, UraoT, IwasakiT, HosokawaD, ShinozakiK. Role of Arabidopsis MYC and MYB homologs in drought- and abscisic acid-regulated gene expression. The Plant Cell. 1997;9(10):1859–68. 10.1105/tpc.9.10.1859 .9368419PMC157027

[7] FinkelsteinRR, LynchTJ. The arabidopsis abscisic acid response gene ABI5 encodes a basic leucine zipper transcription factor. The Plant Cell. 2000;12(4):599–609. .1076024710.1105/tpc.12.4.599PMC139856

[8] MareC, MazzucotelliE, CrosattiC, FranciaE, StancaAM, CattivelliL. Hv-WRKY38: a new transcription factor involved in cold- and drought-response in barley. Plant molecular biology. 2004;55(3):399–416. 10.1007/s11103-004-0906-7 .15604689

[9] SongCP, AgarwalM, OhtaM, GuoY, HalfterU, WangPC, et al Role of an Arabidopsis AP2/EREBP-type transcriptional repressor in abscisic acid and drought stress responses. The Plant Cell. 2005;17(8):2384–96. 10.1105/tpc.105.033043 .15994908PMC1182496

[10] EulgemT. Regulation of the Arabidopsis defense transcriptome. Trends in plant science. 2005;10(2):71–8. 10.1016/j.tplants.2004.12.006 .15708344

[11] GongPJ, ZhangJH, LiHX, YangCX, ZhangCJ, ZhangXH, et al Transcriptional profiles of drought-responsive genes in modulating transcription signal transduction, and biochemical pathways in tomato. Journal of experimental botany. 2010;61(13):3563–75. 10.1093/jxb/erq167 .20643807PMC2921197

[12] RabbaniMA, MaruyamaK, AbeH, KhanMA, KatsuraK, ItoY, et al Monitoring expression profiles of rice genes under cold, drought, and high-salinity stresses and abscisic acid application using cDNA microarray and RNA get-blot analyses. Plant physiology. 2003;133(4):1755–67. 10.1104/pp.103.025742 .14645724PMC300730

[13] TalameV, OzturkNZ, BohnertHJ, TuberosaR. Barley transcript profiles under dehydration shock and drought stress treatments: a comparative analysis. Journal of experimental botany. 2007;58(2):229–40. Epub 2006/11/18. 10.1093/jxb/erl163 .17110587

[14] MiaoWG, WangXB, SongCF, WangY, RenYH, WangJS. Transcriptome analysis of Hpa1(Xoo) transformed cotton revealed constitutive expression of genes in multiple signalling pathways related to disease resistance. Journal of experimental botany. 2010;61(15):4263–75. 10.1093/jxb/erq227 .20667962PMC2955741

[15] Hayano-KanashiroC, Calderon-VazquezC, Ibarra-LacletteE, Herrera-EstrellaL, SimpsonJ. Analysis of Gene Expression and Physiological Responses in Three Mexican Maize Landraces under Drought Stress and Recovery Irrigation. PLoS One. 2009;4(10). ARTN e7531 10.1371/journal.pone.0007531 .19888455PMC2766256

[16] PrattLH, LiangC, ShahM, SunF, WangHM, ReidSP, et al Sorghum expressed sequence tags identify signature genes for drought, pathogenesis, and skotomorphogenesis from a milestone set of 16,801 unique transcripts. Plant physiology. 2005;139(2):869–84. 10.1104/pp.105.066134 .16169961PMC1256002

[17] SekiM, NarusakaM, IshidaJ, NanjoT, FujitaM, OonoY, et al Monitoring the expression profiles of 7000 Arabidopsis genes under drought, cold and high-salinity stresses using a full-length cDNA microarray. Plant journal. 2002;31(3):279–92. 10.1046/j.1365-313X.2002.01359.x .12164808

[18] HuangDQ, WuWR, AbramsSR, CutlerAJ. The relationship of drought-related gene expression in Arabidopsis thaliana to hormonal and environmental factors. Journal of experimental botany. 2008;59(11):2991–3007. 10.1093/jxb/ern155 .18552355PMC2504347

[19] ZongY, SunP, LiuJ, YueXY, NiuQF, TengYW. Chloroplast DNA-based genetic diversity and phylogeography of Pyrus betulaefolia (Rosaceae) in Northern China. Tree Genet Genomes. 2014;10(3):739–49. 10.1007/s11295-014-0718-0

[20] OkuboM, SakurataniT. Effects of sodium chloride on survival and stem elongation of two Asian pear rootstock seedlings. Scientia Horticulturae. 2000;85(1–2):85–90. 10.1016/S0304-4238(99)00141-7

[21] HuangXS, LiKQ, XuXY, YaoZH, JinC, ZhangSL. Genome-wide analysis of WRKY transcription factors in white pear (Pyrus bretschneideri) reveals evolution and patterns under drought stress. BMC genomics. 2015;16(1):1104 Epub 2015/12/26. 10.1186/s12864-015-2233-6 26704366PMC4691019

[22] HuangXS, LiKQ, JinC, ZhangSL. ICE1 of Pyrus ussuriensis functions in cold tolerance by enhancing PuDREBa transcriptional levels through interacting with PuHHP1. Scientific reports. 2015;5 Artn 17620 10.1038/Srep17620 .26626798PMC4667267

[23] QiXX, WuJ, WangLF, LiLT, CaoYF, TianLM, et al Identifying the candidate genes involved in the calyx abscission process of 'Kuerlexiangli' (Pyrus sinkiangensis Yu) by digital transcript abundance measurements. BMC genomics. 2013;14 Artn 727 10.1186/1471-2164-14-727 .24152304PMC4046677

[24] WuJ, WangZW, ShiZB, ZhangS, MingR, ZhuSL, et al The genome of the pear (Pyrus bretschneideri Rehd.). Genome Res. 2013;23(2):396–408. 10.1101/gr.144311.112 .23149293PMC3561880

[25] LiRQ, YuC, LiYR, LamTW, YiuSM, KristiansenK, et al SOAP2: an improved ultrafast tool for short read alignment. Bioinformatics. 2009;25(15):1966–7. 10.1093/bioinformatics/btp336 .19497933

[26] MortazaviA, WilliamsBA, MccueK, SchaefferL, WoldB. Mapping and quantifying mammalian transcriptomes by RNA-Seq. Nature methods. 2008;5(7):621–8. 10.1038/nmeth.1226 I .18516045PMC13303166

[27] AudicS, ClaverieJM. The significance of digital gene expression profiles. Genome Res. 1997;7(10):986–95. .933136910.1101/gr.7.10.986

[28] de HoonMJL, ImotoS, NolanJ, MiyanoS. Open source clustering software. Bioinformatics. 2004;20(9):1453–4. 10.1093/bioinformatics/bth078 .14871861

[29] SaldanhaAJ. Java Treeview-extensible visualization of microarray data. Bioinformatics. 2004;20(17):3246–8. 10.1093/bioinformatics/bth349 .15180930

[30] MulderNJ, ApweilerR, AttwoodTK, BairochA, BarrellD, BatemanA, et al The InterPro Database, 2003 brings increased coverage and new features. Nucleic acids research. 2003;31(1):315–8. 10.1093/nar/gkg046 .12520011PMC165493

[31] ZdobnovEM, ApweilerR. InterProScan—an integration platform for the signature-recognition methods in InterPro. Bioinformatics. 2001;17(9):847–8. 10.1093/bioinformatics/17.9.847 .11590104

[32] HarrisMA, ClarkJ, IrelandA, LomaxJ, AshburnerM, FoulgerR, et al The Gene Ontology (GO) database and informatics resource. Nucleic acids research. 2004;32:D258–D61. 10.1093/nar/gkh036 .14681407PMC308770

[33] YeJ, FangL, ZhengHK, ZhangY, ChenJ, ZhangZJ, et al WEGO: a web tool for plotting GO annotations. Nucleic acids research. 2006;34:W293–W7. 10.1093/nar/gkl1031 .16845012PMC1538768

[34] KanehisaM, GotoS, HattoriM, Aoki-KinoshitaKF, ItohM, KawashimaS, et al From genomics to chemical genomics: new developments in KEGG. Nucleic acids research. 2006;34:D354–D7. 10.1093/nar/gkj102 .16381885PMC1347464

[35] LivakKJ, SchmittgenTD. Analysis of relative gene expression data using real-time quantitative PCR and the 2(T)(-Delta Delta C) method. Methods. 2001;25(4):402–8. 10.1006/meth.2001.1262 .11846609

[36] HuangXS, LiuJH, ChenXJ. Overexpression of PtrABF gene, a bZIP transcription factor isolated from Poncirus trifoliata, enhances dehydration and drought tolerance in tobacco via scavenging ROS and modulating expression of stress-responsive genes. BMC plant biology. 2010;10 Artn 230 10.1186/1471-2229-10-230 .20973995PMC3017851

[37] HuangXS, LuoT, FuXZ, FanQJ, LiuJH. Cloning and molecular characterization of a mitogen-activated protein kinase gene from Poncirus trifoliata whose ectopic expression confers dehydration/drought tolerance in transgenic tobacco. Journal of experimental botany. 2011;62(14):5191–206. 10.1093/jxb/err229 .21778184PMC3193021

[38] Fernandez-CalvoP, ChiniA, Fernandez-BarberoG, ChicoJM, Gimenez-IbanezS, GeerinckJ, et al The Arabidopsis bHLH Transcription Factors MYC3 and MYC4 Are Targets of JAZ Repressors and Act Additively with MYC2 in the Activation of Jasmonate Responses. The Plant cell. 2011;23(2):701–15. 10.1105/tpc.110.080788 .21335373PMC3077776

[39] GortonHL. Water Relations in Pulvini from Samanea-Saman .1. Intact Pulvini. Plant physiology. 1987;83(4):945–50. 10.1104/Pp.83.4.945 .16665369PMC1056480

[40] XuYJ, GaoS, YangYJ, HuangMY, ChengLN, WeiQ, et al Transcriptome sequencing and whole genome expression profiling of chrysanthemum under dehydration stress. BMC genomics. 2013;14 Artn 662 10.1186/1471-2164-14-662 .24074255PMC3849779

[41] WangZ, GersteinM, SnyderM. RNA-Seq: a revolutionary tool for transcriptomics. Nature reviews genetics. 2009;10(1):57–63. 10.1038/nrg2484 I .19015660PMC2949280

[42] BrayEA. Genes commonly regulated by water-deficit stress in Arabidopsis thaliana. Journal of experimental botany. 2004;55(407):2331–41. 10.1093/jxb/erh270 .15448178

[43] HuangXS, WangW, ZhangQ, LiuJH. A Basic Helix-Loop-Helix Transcription Factor, PtrbHLH, of Poncirus trifoliata Confers Cold Tolerance and Modulates Peroxidase-Mediated Scavenging of Hydrogen Peroxide. Plant physiology. 2013;162(2):1178–94. 10.1104/pp.112.210740 .23624854PMC3668048

[44] NingJ, LiXH, HicksLM, XiongLZ. A Raf-Like MAPKKK Gene DSM1 Mediates Drought Resistance through Reactive Oxygen Species Scavenging in Rice. Plant physiology. 2010;152(2):876–90. 10.1104/pp.109.149856 .20007444PMC2815886

[45] MoranoKA. New tricks for an old dog: The evolving world of Hsp70. Annals of the New York Academy of Sciences. 2007;1113:1–14. 10.1196/annals.1391.018 .17513460

[46] DuZ, ZhouX, LingY, ZhangZH, SuZ. agriGO: a GO analysis toolkit for the agricultural community. Nucleic acids research. 2010;38:W64–W70. 10.1093/nar/gkq310 .20435677PMC2896167

[47] LenkaSK, KatiyarA, ChinnusamyV, BansalKC. Comparative analysis of drought-responsive transcriptome in Indica rice genotypes with contrasting drought tolerance. Plant biotechnology journal. 2011;9(3):315–27. 10.1111/j.1467-7652.2010.00560.x .20809928

[48] GuoPG, BaumM, GrandoS, CeccarelliS, BaiGH, LiRH, et al Differentially expressed genes between drought-tolerant and drought-sensitive barley genotypes in response to drought stress during the reproductive stage. Journal of experimental botany. 2009;60(12):3531–44. 10.1093/jxb/erp194 .19561048PMC2724701

[49] ChavesMM, FlexasJ, PinheiroC. Photosynthesis under drought and salt stress: regulation mechanisms from whole plant to cell. Annals of botany. 2009;103(4):551–60. 10.1093/aob/mcn125 .18662937PMC2707345

[50] ChavesM, FlexasJ, PinheiroC. Photosynthesis under drought and salt stress—regulation mechanisms from the whole plant to cell. Photosynthesis research. 2007;91(2–3):300–300.10.1093/aob/mcn125PMC270734518662937

[51] TenaG, AsaiT, ChiuWL, SheenJ. Plant mitogen-activated protein kinase signaling cascades. Current opinion in plant biology. 2001;4(5):392–400. 10.1016/S1369-5266(00)00191-6 .11597496

[52] NakagamiH, PitzschkeA, HirtH. Emerging MAP kinase pathways in plant stress signalling. Trends in plant science. 2005;10(7):339–46. 10.1016/j.tplants.2005.05.009 .15953753

[53] UranoK, MaruyamaK, OgataY, MorishitaY, TakedaM, SakuraiN, et al Characterization of the ABA-regulated global responses to dehydration in Arabidopsis by metabolomics. The Plant journal. 2009;57(6):1065–78. 10.1111/j.1365-313X.2008.03748.x .19036030

[54] ShinozakiK, Yamaguchi-ShinozakiK. Gene networks involved in drought stress response and tolerance. Journal of experimental botany. 2007;58(2):221–7. Epub 2006/11/01. 10.1093/jxb/erl164 .17075077

[55] UmezawaT, OkamotoM, KushiroT, NambaraE, OonoY, SekiM, et al CYP707A3, a major ABA 8'-hydroxylase involved in dehydration and rehydration response in Arabidopsis thaliana. The Plant journal. 2006;46(2):171–82. Epub 2006/04/21. 10.1111/j.1365-313X.2006.02683.x .16623881

[56] ColebrookEH, ThomasSG, PhillipsAL, HeddenP. The role of gibberellin signalling in plant responses to abiotic stress. Journal of experimental biology. 2014;217(Pt 1):67–75. Epub 2013/12/20. 10.1242/jeb.089938 .24353205

[57] FujiiH, VersluesPE, ZhuJK. Arabidopsis decuple mutant reveals the importance of SnRK2 kinases in osmotic stress responses in vivo. Proceedings of the National Academy of Sciences of the United States of America. 2011;108(4):1717–22. 10.1073/pnas.1018367108 .21220313PMC3029766

[58] SharpRE, LeNobleME. ABA, ethylene and the control of shoot and root growth under water stress. Journal of experimental botany. 2002;53(366):33–7. 10.1093/jexbot/53.366.33 .11741038

[59] FujiiH, ChinnusamyV, RodriguesA, RubioS, AntoniR, ParkSY, et al In vitro reconstitution of an abscisic acid signalling pathway. Nature. 2009;462(7273):660–U138. 10.1038/nature08599 .19924127PMC2803041

[60] BoudsocqM, DroillardMJ, Barbier-BrygooH, LauriereC. Different phosphorylation mechanisms are involved in the activation of sucrose non-fermenting 1 related protein kinases 2 by osmotic stresses and abscisic acid. Plant molecular biology. 2007;63(4):491–503. 10.1007/s11103-006-9103-1 .17103012

[61] BrayEA. Genes commonly regulated by water-deficit stress in Arabidopsis thaliana. Journal of experimental botany. 2004;55(407):2331–41. Epub 2004/09/28. 10.1093/jxb/erh270 .15448178

[62] LiuJH, PengT, DaiWS. Critical cis-Acting Elements and Interacting Transcription Factors: Key Players Associated with Abiotic Stress Responses in Plants. Plant molecular biology reporter. 2014;32(2):303–17. 10.1007/s11105-013-0667-z

[63] HuHH, DaiMQ, YaoJL, XiaoBZ, LiXH, ZhangQF, et al Overexpressing a NAM, ATAF, and CUC (NAC) transcription factor enhances drought resistance and salt tolerance in rice. Proceedings of the National Academy of Sciences of the United States of America. 2006;103(35):12987–92. 10.1073/pnas.0604882103 .16924117PMC1559740

[64] AbeH, UraoT, ItoT, SekiM, ShinozakiK, Yamaguchi-ShinozakiK. Arbaidopsis AtMYC2 (bHLH) and AtMYB2 (MYB) function as transcriptional activators in abscisic acid signaling. The Plant cell. 2003;15(1):63–78. 10.1105/tpc.006130 .12509522PMC143451

[65] CominelliE, GalbiatiM, VavasseurA, ContiL, SalaT, VuylstekeM, et al A guard-cell-specific MYB transcription factor regulates stomatal movements and plant drought tolerance. Current biology. 2005;15(13):1196–200. 10.1016/j.cub.2005.05.048 .16005291

[66] LiHM, SunJQ, XuYX, JiangHL, WuXY, LiCY. The bHLH-type transcription factor AtAIB positively regulates ABA response in Arabidopsis. Plant molecular biology. 2007;65(5):655–65. 10.1007/s11103-007-9230-3 .17828375

[67] ZouXL, ShenQJX, NeumanD. An ABA inducible WRKY gene integrates responses of creosote bush (Larrea tridentata) to elevated CO2 and abiotic stresses. Plant Science. 2007;172(5):997–1004. 10.1016/j.plantsci.2007.02.003

[68] WeiW, ZhangYX, HanL, GuanZQ, ChaiTY. A novel WRKY transcriptional factor from Thlaspi caerulescens negatively regulates the osmotic stress tolerance of transgenic tobacco. Plant cell reports. 2008;27(4):795–803. 10.1007/s00299-007-0499-0 .18183400

[69] ZhengXN, ChenB, LuGJ, HanB. Overexpression of a NAC transcription factor enhances rice drought and salt tolerance. Biochemical and biophysical research communications. 2009;379(4):985–9. 10.1016/j.bbrc.2008.12.163 .19135985

[70] StorozhenkoS, De PauwP, Van MontaguM, InzeD, KushnirS. The heat-shock element is a functional component of the Arabidopsis APX1 gene promoter. Plant physiology. 1998;118(3):1005–14. 10.1104/pp.118.3.1005 .9808745PMC34773

[71] WangWX, VinocurB, ShoseyovO, AltmanA. Role of plant heat-shock proteins and molecular chaperones in the abiotic stress response. Trends in plant science. 2004;9(5):244–52. 10.1016/j.tplants.2004.03.006 .15130550

[72] RongW, QiL, WangAY, YeXG, DuLP, LiangHX, et al The ERF transcription factor TaERF3 promotes tolerance to salt and drought stresses in wheat. Plant biotechnology journal. 2014;12(4):468–79. 10.1111/pbi.12153 .24393105

[73] HaninM, BriniF, EbelC, TodaY, TakedaS, MasmoudiK. Plant dehydrins and stress tolerance: versatile proteins for complex mechanisms. Plant signaling & behavior. 2011;6(10):1503–9. Epub 2011/09/08. 10.4161/psb.6.10.17088 .21897131PMC3256378

[74] HuangY, LiMY, WangF, XuZS, HuangW, WangGL, et al Heat shock factors in carrot: genome-wide identification, classification, and expression profiles response to abiotic stress. Molecular biology reports. 2015;42(5):893–905. 10.1007/s11033-014-3826-x .25403331

